RETRACTED

# MicroRNA-424 Is Down-Regulated in Hepatocellular Carcinoma and Suppresses Cell Migration and Invasion through c-Myb

**DOI:** 10.1371/journal.pone.0091661

**Published:** 2014-03-27

**Authors:** Lei Yu, Guo-feng Ding, Changzhi He, Lei Sun, YanFang Jiang, Liying Zhu

**Affiliations:** 1 Department of Infectious Disease, The Fourth Hospital of Harbin Medical University, Harbin, Heilongjiang, China; 2 Department of Infectious Disease, Binzhou Medical University Hospital, Binzhou, Shandong, China; 3 The Graduate School of Harbin Medical University, Harbin, Heilongjiang, China; 4 Department of Ophthalmology, The Fourth Hospital of Harbin Medical University, Harbin, Heilongjiang, China; 5 Key Laboratory of Zoonosis Research, Ministry of Education, Institute of Zoonosis, Jilin University, Changchun, Jilin, China; Department of Central Laboratory, the Second Part of First Hospital, Jilin University, Changchun, Jilin, China; The University of Hong Kong, China

## Abstract

Hepatocellular carcinoma (HCC) is one of the leading causes of cancer-related mortality worldwide. MicroRNAs (miRNAs) are important regulators of multiple cellular processes, and the aberrant miRNAs expressions have been observed in different types of cancer including HCC. Their pathysiologic role and their relevance to tumorigenesis are still largely unknown. In this study, we demonstrated the down-regulation of miR-424 in HCC cell lines and tissues by quantitative RT-PCR analyses. Overexpression of miR-424 reduced the HCC cell prolifetation, migration, and invasion. Conversely, inhibiton of miR-424 expression significantly accelerated the cell proliferation, migration, and invasion. In addition, we further identified c-Myb as a functional downstream target of miR-424 by directly targeting the 3′UTR of c-Myb. Furthermore, overexpression of c-Myb impaired miR-424-induced inhibition of proliferation and invasion in HCC cells. Our results demonstrated that miR-424 was involved in tumorigenesis of HCC at least in part by suppression of c-Myb.

## Introduction

Hepatocellular carcinoma (HCC) is the sixth most prevalent cancer wordwide and the fourth most common cause of death from cancer; the highest age-standardized mortality rate is in China, which alone accounts for 53% of all liver cancer deaths worldwide [1], [2]. Due to the difficulty of effectively diagnosing HCC at its early stage, only about 10 to 20% of patients with HCC are currently eligible for surgical treatment [3], [4]. Therefore, it is necessary to elucidate the molecular mechanisms involved in HCC in order to identify novel markers for diagnosis, prognosis, and treatment for patients with this disease.

microRNAs (miRNAs) are evolutionarily conserved, endogenous, single-stranded, non-coding RNA molecules with an important role in regulation of gene post-transcriptionally expression [5], [6]. miRNAs play critical roles in several biological processes involving cell proliferation, differentiation, apoptosis, and stress resistance [7]. Studies have revealed that aberrant miRNA expression has been associated with the development and progression of a variety of cancers, including HCC [8]–[10]. For example, miR-21, miR-181b, miR-221, miR-222, and miR-122 are upregulated in HCC tumor tissues compared with nontumor tissues [11]–[16]. These findings suggest that miRNAs could be utilized as biomakers for diagnosis and prognosis prediction of cancers [17]–[19]. Furthermore, miRNAs can have tumor suppressor or oncogenic characteristics. However, there still remains a lot to understand as regards the involvement of miRNAs in hepatocarcinogenesis and progression of HCC.

RETRACTED

In the current study, we found that miR-424 was down-regulated in HCC cell lines and primary tumor samples, and miR-424 was further identified to be a tumor suppressor, as restoration of miR-424 expression in HCC cell lines could reduce cell proliferation and suppressed cell migration and invasion. Additionally, c-Myb, an important pro-invasive molecule, was identified to be a direct target of miR-424, and the proinvasion function of miR-424 is further suggested to be mainly through targeting c-Myb expression. Thus, our data suggest important roles of miR-424 in HCC pathogenesis and indicate its potential application in cancer therapy.

## Results

### miR-424 was down-regulated in HCC tissue and cells

To validate the tumor suppressor role of miR-424 in clinical hepatoma, we analyzed the expression of miR-424 in 80 pairs of clinical HCCs and adjacent nontumorous liver tissues and cell lines. The expression of miR-424 in HCC cells lines (HepG2, Hep3B, Bel7402, SMMC-7721) exhibited low expression compared to the normal hepatocytes (HL-7792 cells) (Fig. 1A). miR-424 was down-regulated in 68 cases (68/80, 85%) compared with adjacent tissues. (Fig. 1B). In general, the expression of miR-424 in HCC tissues was significant lower than in adjacent tissues. (Fig. 1C, p<0.001) Moreover, low levels of miR-424 expression were associated with pTNM stage (p = <0.01, stage I vs. III, p = 0. <0.01, stage II vs. IV) (Fig. 1D), and even lower levels of miR-424 were associated with pM stage (p = <0.01, metastasis vs. no metastasis) in HCC patients (Fig. 1E). These data suggested that alterations of miR-424 could be involved in HCC progression.

**Figure 1:** The expression of miR-424 is down-regulated in both primary HCC tissuess and cell lines. (A) qRT-PCR analysis of miR-424 expression in normal hepatopcytes (HL-7792 cells) and HCC cells (HepG2, Hep3B, Bel7402, SMMC-7721). (B) qRT-PCR analysis of miR-424 expression in 80 pairs HCC tissues and their corresponding adjacent nontumorous livers. The expression of miR-424 was normalized to U6 snRNA. (C) Relative miR-424 expression levels in HCC tissues and adjacent normal regions; (D) and (E) Statistical analysis of the association between miRNA level, pTNM stage (I, II, III and IV) and pM stage (No metastasis and Metastasis, respectively); *p<0.05, and **p<0.01.

RETRACTED

### miR-424 inhibited HCC cell proliferation and Ki-67 expression

HCC cells were transfected with scrambled control oligo or miR-424 mimics and inhibitors, which exhibited a high transfection efficiency (Fig. 2A). CCK-8 proliferation assay results showed that cell proliferation was inhibited in miR-424 mimic-transfected HCC cells compared with scrambled oligo-transfected cells or untreated cells (Fig. 2B). The proliferative effect of miR-424 was further confirmed by evaluating Ki-67 expression. As shown in Fig. 2C and D, there was a significant decrease in the protein and mRNA levels of Ki-67 in the group transfected with miR-424 mimics when compared with the control or untreated group. Conversely, miR-424 inhibitor significantly accelerated the cell proliferation and Ki-67 expression of HCC cells.

**Figure 2:** Overexpression of miR-424 inhibits the cell proliferation in HepG2. (A) qRT-PCR analysis of miR-424 expression after the transfection of miR-424 mimics, inhibitors or scramble or no transfection. (B) The CCK8 assay used to evalute the proliferation of HepG2 cells after transfection with the miR-424 mimics, inhibitors or scramble or no transfection. (C) (C) miR-424 inhibited Ki-67 mRNA expression. HepG2 cells were transfected with miR-424 mimics, inhibitors or scramble or no transfection. Ki-67 mRNA levels were detected by real-time PCR. The expression of Ki-67 was normalized to GAPDH. (D) miR-424 inhibited Ki-67 protein expression. HepG2 cells were transfected with miR-424 mimics, inhibitors or scramble or no transfection. Ki-67 levels were detected by western blot. GAPDH was also detected as a loading control. Values are presented as the mean ± SD. Compared with control, *p<0.05, ** p<0.01, and ***p<0.001.

### miR-424 inhibited HCC cell migration and invasion in vitro

These cells treated with miR-424 mimics were distinctively less migratory than scrambled control or untreated cells at 24, and 36 hours after scratching (Fig. 3A). Conversely, miR-424 inhibitor significantly increased the cell migration of HepG2. Furthermore, we conducted cell invasion assay of Matrigel and stained the invaded cells to measure the directional invasion ability of the cells after ectopically expressing miR-424 in HepG2 cells. The invasiveness of cells transfected with miR-424 mimics was dramatically decreased compared with the scrambled control and untreated cells. However, miR-424 inhibitor significantly increased the cell invasion of HepG2. (Fig. 3B)

**Figure 3:** Ectopic expression of miR-424 suppressed HCC cell migration and invasion. (A) Wound healing assays of HepG2 cells after treatment with miRNA mimics, inhibitors or scramble or no transfection; the relative ratio of wound closure per field is shown. (B) Transwell analysis of HepG2 cells after treatment with miRNA mimics, inhibitors or scramble or no transfection; the relative ratio of invasive cells per field is shown below, ** p<0.01, and ***p<0.001.

RETRACTED

### miR-424 targeted at c-Myb

As predicted by TargetScan, there was complementarity between hsa-miR-424 and c-Myb 3′-UTR (Fig. 4A). The effect of miR-424 on the translation of c-Myb mRNA into protein was assessed by luciferase reporter assay in HCC cells (Fig. 5B). The overexpression of miR-424 remarkably reduced luciferase activity in the c-Myb wild-type reporter gene but not the mutant c-Myb 3′UTR, indicating that miR-424 directly targeted the c-Myb 3′UTR. To assess the regulation of miR-424 in c-Myb expression, the protein and mRNA level of c-Myb was analyzed after miR-424 overexpression. C-Myb protein but not mRNA was obviously decreased in the presence of miR-424 mimics compared with the scrambled control in both HepG2 cells (Fig. 4C, D, and E).

**Figure 4:** miR-424 targets at c-Myb in HCC cells. (A) The sequences of miR-424 binding sites within the human c-Myb 3′UTRs and schematic reporter constructs, in this panel, c-Myb-WT represent the reporter constructs containing the entire 3′UTR sequences of c-Myb. C-Myb-MUT represent the reporter constructs containing mutated nucleotides. (B) The analysis of the relative luciferase activities of c-Myb-WT, c-Myb-MUT in 293T cells. The error bars are derived from triplicate expriments. (C) qRT-PCR analysis of c-Myb mRNA expression in HepG2 cells after treatment with miRNA mimics or scramble or no transfection. The expression of c-Myb was normalized to GAPDH. (D) (E) Western blot analysis of c-Myb expression in HepG2 cells transfected with miR-424 mimics or scramble or no transfection. GAPDH was also detected as a loading control. ** p<0.01.

**Figure 5:** Overexpression of c-Myb impairs miR-424-induced inhibition of proliferation and invasion in HCC cells. (A) Western blot analysis of c-Myb expression in 8 miR-424 down-regulated HCC tissues. GAPDH was also detected as a loading control. (B) Western blot analysis of c-Myb expression in HepG2 cells co-transfected with either miR-424 mimics or scramble and pCDNA-c-Myb or pCDNA empty vector; GAPDH was also detected as a loading control. (C) Cell growth curves in HepG2 cells transfected with different combinations. (D) Transwell analysis of HepG2 cells treated with different combinations. The relative ratio of invasive cells per field is shown right. *p<0.05,** p<0.01, ***p<0.001.

RETRACTED

### Overexpression of c-Myb impaired miR-424-induced inhibition of proliferation and invasion in HCC cells

To assess the regulation of miR-424 in c-Myb expression, the protein level of c-Myb was analyzed in eight miR-424 down-regulated HCC tissues. c-Myb was up-regulated in all HCC tissues. (Fig. 5A) Next, we adapted a “rescue” strategy in order to examine the functional relevance of the miR-424/c-Myb interaction in HCC cells. The level of c-Myb was reduced when miR-424 mimic were transfected after 24 h treatment of pcDNA-c-Myb (Fig. 5B). In agreement with the reduced expression of target proteins, decreased cell proliferation (Fig. 5C), accompanied by decreased cell invasion (Fig. 5D) were also observed in HCC cells transfected with miR-424 mimic following treatment of pcDNA-c-Myb construct. Thus, we concluded that the repression of cell growth by miR-424 is typically the consequence of decreased c-Myb expression in HCC.

## Discussion

HCC is a primary neoplasm of the liver and the fourth most common cause of death from cancer worldwide [21]. However, its underlying molecular mechanism remains largely unknown. Growing evidence has suggested that dysregulation of miRNAs may contribute to tumorigesis [22]. Thus, miRNAs are increasingly viewed as a potential diagnostic and therapeutic tool. In our study, we analyzed the expression of miR-424 in 80 HCC patients and HCC cell lines found that miR-424 expression is down-regulated in HCC cells lines and tissues compared with paired adjacent nontumoral tissues. Statistical analyses reveal that the expression level of miR-424 was significantly correlated with metastasis. In addition, we found that restored expression miR-424 suppressed HCC cell proliferation, migration and invasion in HCC cells HepG2. Moreover, we also identified c-Myb as a direct target of miR-424. Our findings, together with those other groups, suggest that miR-424 has a fundamental role in HCC tumorigenesis and cancer cell proliferation and invasion.

Previous studies have shown that miR-424 may act as a potential suppressor miRNA [23], [24]. For example, miR-424 was down-regulated in cervical cancer tissues and correlated with progression of the cervical cancer [25]. miR-424 inhibited cervical cancer cells proliferation, migration and invasion. Furthermore, a decreased aberrant miR-424 expression is also accompanied by a potent suppression of oncogene PLAG1 in chronic lymphocytic leukemia [26], [27]. In line with these results, miR-424 was also found to be commonly deregulated in hepatocellular adenoma (HCA) from type I glycogen storage disease (GSD I) and general population HCA [28]. However, their expression and function in HCC remains to be determined. Consistent with these previous studies,our study has found that miR-424 was down-regulated in 68 cases (68/80, 85%) HCC tissues compared with the adjacent tissues and the expression of miR-424 in HCC tissues was significantly lower than in adjacent tissues. We also found that the lower expression of miR-424 in HCC specimens was correlated with metastasis. All of these evidences indicated that miR-424 might contribute to HCC malignancy.

RETRACTED

To elucidate the role of miR-424 in the development of HCC, cell transfection was done. Overexpression of miR-424 significantly suppressed HCC cell proliferation, invasion and migration, indicating that repression of miR-424 might induce tumor development and progression in HCC carcinogenesis. These results indicated that miR-424 may act as a tumor-suppressor whose downregulation may contribute to the progression and metastasis of HCC.

To explore the molecular mechanism by which miR-424 suppressed HCC cell line growth, migration and invasion, we identified c-Myb as a direct target of miR-424 in HCC cells, and this conclusion is supported by the following reasons: complementary sequence of miR-424 was identified in the 3′UTR of c-Myb mRNA; ectopic of miR-424 led to a significant reduction in c-Myb at the protein level; overexpression of miR-424 inhibited c-Myb 3′UTR luciferase report activity and this effect was abolished by mutation of the miR-424 seed binding site. This result is line with the previous study that miR-424 restrained c-Myb in Epstein-Barr virus-associated B-cell lymphoma [29]. These results indicate that miR-424 may function as a tumor suppressor partly mediated by repressing c-Myb expression in HCC development.

The Myb protein was first identified as an oncogene that causes leukemia in chickens in 1979 [30], [31]. As a prototype oncogene, c-Myb is overexpressed in a number of human cancers, and its overexpression contributes to malignant transformation by regulating the expression of a number of genes participating in multiple aspects of tumorigenesis, such as cell growth, angiogenesis, and resistance to apoptosis [32]–[34]. Furthermore, overexpression of c-Myb is considered to be a new potential or even an independent predictor of poor prognosis for clinical patients in multiple types of cancer [35]–[37]. Previous studies have shown that c-Myb mRNA expression was up-regulated in HCC compared with adjacent pair-matched non-tumor tissues and survival analysis indicated that strong c-Myb expression had lower disease-specific survival rates than those with negative c-Myb expression [38]–[40]. However, the underlying mechanisms are unclear. Our data showed that the ability of miR-424 to target c-Myb may provide one such mechanism of post-transcriptional control of c-Myb.

RETRACTED

In conclusion, the data presented here strongly suggest that miR-424 acts as a tumor suppressor in HCC. Our study showed that miR-424 is significantly down-expressed in HCC cell lines and clinical specimens and reintroduction of miR-424 in HCC cells inhibited cell growth, suppressed cell invasion and migration partly through suppressing the c-Myb. This finding not only helps us to understand the molecular mechanism of HCC carcinogenesis, but also gives us a strong rationale to further investigate miR-424 may as a potential biomaker and therapeutic target for HCC.

## Materials and Methods

### Ethics statement

All patients agreed to participate in the study and gave written informed consent. This study was approved by the ethical board of the institute of The Fourth Hospital of Harbin Medical University and complied with Declaration of Helsinki.

### Samples and cases

HCC and their morphologically normal tissues (located >3 cm away from the tumor) were obtained between 2009 and 2012 from 80 HCC patients undergoing surgery at The Fourth Hospital of Harbin Medical University. Tissue samples were cut into two parts, one was fixed with 10% formalin for histopathological diagnosis, and the other was immediately snap-frozen in liquid nitrogen, and stored in liquid nitrogen until RNA extraction. None of the patients received radiotherapy or chemotherapy before surgery. The characteristics of patients are described in Table S1 in File S1.

### Cell lines and cell culture

The following human cell lines were used in this study: HepG2, Hep3B, Bel7402, SMMC-7721 and HL-7702. All of these cell lines were purchased from American Type Culture Collection (ATCC, Mannasas,VA, USA). These cells were culture and maintained at RPMI 1640 medium (PAA) supplemented with 10% FBS (GIBCO, NY, USA). Cells were maintained at 37°C in a humidified chamber with 95% air and 5% CO_2_.

### Cell transfection

The miR-424 mimics, miR-424 inhibitor and the scramble mimics were synthesized by GenePharma (Shanghai, China) and transfected into the cells to a final oligonucleotide concentration of 20 nmol/L. All cell transfections were introduced by DharmaFECT1 Reagent (Dharmacon, TX, USA) according to the manufacturer's instructions. For each cell transfection, three replication experiments were performed.

RETRACTED

### Quantitative Real Time RT-PCR

Total RNA was extracted from the cell lines and frozen tumor specimens with Trizol reagent (Invitrogen, Calsbad, CA, USA). The RNA was quantified by assessing its absorbance at 260 nm. The cDNA was synthesized from 2 μg of total RNA using M-MLV reverse transcriptase (Invitrogen). As described by Yu [20], stem-loop RT primers were used for the reverse transcription of miRNAs. MicroRNAs were quantitated by real-time PCR using TaqMan MicroRNA assay (Invitrogen, USA). Real-time PCR was performed using a standard TaqMan PCR protocol. The 20 μl PCRs reactions included 1 μl of RT product, 1 Universal TaqMan Master Mix and 1xTaqMan probe/primer mix (Invitrogen, USA, Table S2 in File S1). For miRNAs, U6 snRNA was used as the endogenous control.

### Cell proliferation assay

Cell proliferation was measured using Cell Counting Kit-8 (Dojindo, Kumamoto, Japan).In accordance with the manufacturer's instructions for Cell Counting Kit-8, harvested cells were seeded in 96-well plates at 1×10^3^ per well (n = 5 for each time point) in a final volume of 100 μL. Cells were cultured for 24, 48, 72, and 96 hours after transfection. CCK-8 solution (10 μL) was added into each well, and the absorbance at 450 nm was measured after incubation for 2 hours at 37°C to calculate the number of viable cells.

### Cell migration and invasion assays

Transfected cells were seeded in 24-well plates. The cell layer was scratched with the tip of a 200 μL pipette. The healing process was observed for 24 and 48 hours. The wound width was measured 24 and 48 hours after scratching in order to evaluate the wound healing ability of tested cells.

Invasion assay was evaluated by the ability of cells passing through Matrigel-coated membrane matrix (BD Biosciences). Cells were seeded onto a Matrigel-coated membrane matrix present in the insert of a 24-well culture plate 24 hours after transfection. Fetal bovine serum was added to the noninvading cells were removed. Invasive cells located on the lower surface of the chamber were stained with 0.1% crystal violet (Sigma) and counted.

### Dual luciferase assays

The 3′ UTRs of c-Myb containing the predicted binding sites of miR-424 were amplified by PCR from human cDNA using primers, and inserted into the pMIR-REPORT luciferase reporter vectors (Ambion, Austin, TX, USA) to get the constructs containing the wild-type c-Myb 3′UTR (c-Myb-WT), c-Myb-MUT contained the sequences with mutations in the first putative binding site of c-Myb 3′UTR. Mutations of the predicted seed regions in these mRNA sequences were created using the primers including the mutated sequences. The recombination constructs, pRL-TK (Promega, WI, USA) and miR-424 or control mimic were co-transfected into 293T cells using lipofectamine 2000 (Invitrogen, Carlsbad, CA, USA). The plasmid of pRL-TK containing Renilla luciferase was used as internal control. Firefly and Renilla luciferase activity were measured using Dual Luciferase Assay (Promega) according to the manufacturer's instructions at 24 h after transfection. All transfection assays were carried out in triplicate.

RETRACTED

### Western blotting analysis

Western blot analysis was performed using standard methods. Proteins were separated on 10% SDS-PAGE, and then transferred to PVDF membranes (Amersham, Buckinghamshire, UK). Membranes were blocked for 2 h with 5% non-fat dried milk and incubated overnight with anti-Ki-67 antibody or anti-c-Myb antibody (Abcam, England) at 1∶1000 dilution; anti-GAPDH antibody (Proteintech,Chicago, USA) at 1∶50,000 dilution. After washing with TBST (10 mM Tris, pH 8.0, 150 mM NaCl, and 0.1% Tween20), the membranes were incubated for 2 h with goat anti-rabbit antibody (zsgb-bio, Beijing, China) at 1∶5000 dilution and 1∶50000 dilution.

### Statistical analysis

Each experiment was performed at least three times. Statistical analysis was performed using SPSS 15.0. Data are presented as the mean ± standard deviation. Statistical analyses were done by analysis of variance (ANOVA) or Student's t test and statistical significance level was set at α = 0.05 (two-side)

## Supporting Information

File S1 **Supporting Information Tables.** Table S1, Clinicopathologic charateristics of patients with HCC. Table S2, Primer sequence.
(DOC)
